This article has been retracted.

# Study of the Structure and Properties of ZnS Utilized in a Fluorescence Biosensor

**DOI:** 10.1155/2021/7067146

**Published:** 2021-08-28

**Authors:** Y. Ren, H. Zhou, X. Wang, Q. W. Liu, X. D. Hou, G. F. Zhang

**Affiliations:** ^1^Henan University of Technology, School of Materials Science and Engineering, Engineering Laboratory of High Temperature Resistance-Wear Materials, Zhengzhou 450007, China; ^2^Key Laboratory of Materials Modification by Laser, Ion and Electron Beams (Ministry of Education), School of Materials Science and Engineering, Dalian University of Technology, Dalian, 116024 Liaoning Province, China

## Abstract

ZnS materials have been widely used in fluorescence biosensors to characterize different types of stem cells due to their excellent fluorescence effect. In this study, ZnS was prepared by vulcanizing nano-Zn particles synthesized using a DC arc plasma. The composition and structure of the ZnS materials were studied by X-ray diffraction (XRD), and their functional group information and optical properties were investigated by using IR spectrophotometry and UV-vis spectrophotometry. It has been found that the synthesized materials consist of Zn, cubic ZnS, and hexagonal ZnS according to the vulcanization parameters. Crystalline ZnS was gradually transformed from a cubic to a hexagonal structure, and the cycling properties first increase, then decrease with increasing sulfurization temperature. There is an optimal curing temperature giving the best cycling performance and specific capacity: the material sulfurized thereat mainly consists of cubic *β*-ZnS phase with a small quantity of Zn and hexagonal *α*-ZnS. The cubic phase ZnS has better conductivity than hexagonal ZnS, as evinced by electrochemical impedance spectroscopy (EIS). The ZnS (as prepared) shows board absorption, which can be used in fluorescence biosensors in cell imaging systems.

## 1. Introduction

Fluorescence biosensors are used in qualitative or quantitative analysis by fluorescence enhancement, quenching, or shift of emission wavelength by fluorescence signals; they are used for cell imaging, so organic fluorescent dyes have been developed, including fluorescein, rhodamine, and coumarin. [1, 2] Compared with these traditional organic fluorescent dyes, ZnS nanomaterials, as important II-VI compound semiconductors, have attracted much attention. Its band gap at room temperature is 3.66 eV, resulting in excellent fluorescence and electroluminescence function, making it a good fluorescent host material.

ZnS quantum dots (QDs) have been developed as promising materials for different uses in devices such as chemical sensors [3], in antibacterial applications, [4] and biological imaging and diagnosis [5–9]. Furthermore, ZnS nanomaterials can be thought of as candidate anode materials of lithium-ion batteries, replacing graphite carbon materials [10]. The performance of lithium-ion batteries depends largely on anode materials [11, 12]. The anode performance, moreover, will deteriorate due to the large volume changes before and after lithium intercalation. Solvothermal synthesis and microwave synthesis are the main methods used to prepare ZnS [13–17]. As a solution, carbon-coated ZnS has been prepared by the solvothermal method in recent years [18]. To prepare ZnS with excellent performance, the new synthetic methods at low cost, with high yield, good stability, and effective elimination of surface defects need to be explored.

In the present work, a simple and low-cost method was used to synthesize ZnS nanomaterials. Firstly, Zn powders were prepared by DC arc plasma and then vulcanized to form ZnS [19]. The advantage therein is that the degree of vulcanizing and the structure of ZnS can be controlled by altering various vulcanizing parameters. Whether it is used as a fluorescent probe or anode material, we are trying to obtain high-performance ZnS materials in terms of their optical and electrochemical properties. The electrochemical properties can be improved and are superior to those of pure Zn or ZnS materials [20].

## 2. Experiments

In a DC arc-discharge plasma evaporation system, the arc was maintained between the bulk Zn (99.99%) anode and the W cathode for 5 min at a current of about 50 A using argon at 0.03 MPa and hydrogen at 0.01 MPa as the carrier gas. After cooling for 120 min and then allowing inflow of air at 0.025 MPa to deactivate the system for 12 h, the vacuum chamber was opened to collect the resulting Zn powder. The uniform mixture of precursors and sublimated sulfur in the ratio of 1 : 1 was put in a closed reactor located at the flat-temperature zone of a tube-type vacuum furnace. The mixture was heated at 200, 250, 300, and 350°C, respectively, at a rate of 10°C/min, then maintained thereat for 2 h. After cooling to room temperature in the furnace, the reactant was dispersed in a porcelain boat and reheated to 200°C for 2 h to remove the remaining sulfur. Finally, the ZnS powders were obtained.

SEM and energy-dispersive X-ray spectrometry (EDX) were used to assess the surface morphology and composition of the ZnS powders (FEI inspect F50). The structure of the ZnS materials was characterized by an XRD-6000 diffractometer with a scanning rate of 4°/min. Functional group information was acquired from Fourier-transform infrared spectroscopy (FTIR, Prestige-21). The optical absorbance was measured on a UV-vis spectrophotometer (SHIMADZU UV-2600i). The electrochemical performance was evaluated using CR2025 coin-type half cells. The anode active material was mixed with conductive additive (Ketjen black) and binder (poly(acrylic acid) (PAA)) in a mass ratio of 8 : 1 : 1. A homogeneous slurry was formed by stirring and dissolving an appropriate amount of deionized water in the mixture. The slurry was uniformly coated onto a copper foil current collector. After drying at 70°C for 12 h and suppressing the reaction, an electrode disk (14 mm in diameter) was obtained with a mass loading of 0.8 mg/cm^2^. The CR2025 button cells were assembled in an argon-filled glovebox using lithium metal as counter electrode. The separator and electrolyte were a microporous polypropylene film and 1 M LiPF_6_ solution in ethylene carbonate (EC)/diethyl carbonate (DEC) (1 : 1 by volume), respectively. The galvanostatic charge-discharge and rate capability were carried out using a Land CT2001A testing system in a voltage window of 0.01–3 V vs. Li/Li+. The cyclic voltammogram (CV) curves were obtained using a CHI660E electrochemical workstation at a scanning rate of 0.1 mV s^–1^ between 0.01 and 3 V. The electrochemical impedance spectroscopy (EIS) analysis was conducted over the frequency range from 0.01 to 100 kHz at an amplitude of 0.5 mV.

## 3. Results and Discussion

The morphology of the ZnS powders was examined using an SEM, as shown in Figure 1. It was observed that powders with different sizes and irregular shapes consisted of smaller particles (<100 nm) and nanosheets (~200 nm) indicated by boxes in Figure 1(a). The EDX spectra evinced the chemical composition of the synthesized powders as mainly composed of zinc and sulfur (Figure 1(b)).

The XRD spectra of the ZnS materials under various sulfurization temperatures are shown in Figure 2. It was found that there were three phases of Zn, *β*-ZnS, and *α*-ZnS in the vulcanization products. Diffraction peaks located at 36.1°, 38.9°, and 43.1° are assigned to the (002), (010), and (011) planes of Zn, at 28.6°, 47.5°, and 56.3° to (111), (220), and (101) of cubic *β*-ZnS, and at 26.9°, 28.5°, and 30.6° to (100), (002), and (011) of hexagonal *α*-ZnS, respectively.

The intensity of Zn diffraction peaks gradually decreased with increasing sulfurization temperature and the Zn diffraction peak disappeared at about 350°C. Moreover, cubic *β*-ZnS had begun to form at 200°C. The main product was cubic *β*-ZnS between 250 and 300°C: this became hexagonal *α*-ZnS at 350°C. It is noteworthy that the phase transformation temperature from *β*-ZnS to *α*-ZnS was greater than 1000°C [12], which indicates that the high surface energy of the Zn nanoparticles plays an important role in the sulfurization process [21].

In the FTIR spectra of the ZnS materials at different sulfurization temperatures as shown in Figure 3(a), the absorption peaks occur at about 3462 cm^−1^ and 1637 cm^−1^, which can be ascribed to the stretching and bending vibration of the O-H and H-O-H bands from external surface water molecules, respectively. [22, 23] Another absorption peak appears at 604 cm^−1^ when the sulfurization temperature increases from 200°C to 300°C. The characteristic vibration of ZnS was observed at 669 or 642 cm^−1^, which was confirmed in Ref.[23, 24] However, with increasing the sulfurization temperature to 350°C, the sharper peak located at 1385 cm^−1^ could be indexed to the stretching vibration of C-O-C bonds. [22] In this study, the excellent optical characteristics of ZnS nanoparticles were observed by absorption spectra. The UV absorption spectrum of ZnS at the sulfurization temperature of 350°C is shown in Figure 3(b): ZnS nanoparticles had a wider range of absorption and show a peak corresponding to 1s-1s electronic transitions therein [22]. The absorption peak position of ZnS was 313 nm, but the maximum absorbance cut-off wavelength was observed at about 500 nm (albeit weak).

At a constant current density of 0.5 A/g, the charge/discharge tests of the cells assembled from the ZnS materials prepared at various sulfurization temperatures were conducted (Table 1). With increasing sulfurization temperature, the first discharge capacity increases from 527.8 to 1052.0 mAh/g and first charge capacity from 405.3 to 511.6 mAh/g. Unexceptionally, the capacity of all such cells decreases with increased cycling. The discharge capacity retention ratio after 300 cycles increases slowly with increasing sulfurization temperature, reaching a maximum of 23.1% at 300°C, and then falling to 9.2%. Under same conditions, the discharge capacity retention ratio of the pure Zn is only 15.4% after 100 cycles: the cycling performance of the Zn/ZnS composites is superior to that of Zn or ZnS. Two main reasons for this are the volumetric expansion of the ZnS materials and the shuttle effects of the elemental S therein; moreover, these two reasons act in mutual opposition. The first factor dominates under lower sulfurization, and the second at higher degrees of vulcanizing, which leads to the existence of an optimal cycle performance.

The rate capability of the ZnS materials was measured in a range of charge/discharge current density 0.1-1.0 A/g. As shown in Figure 4(a), the current density was changed every five cycles. The average specific capacity on each stage for different samples is illustrated in Figure 4(b): the rate capability of samples presents stepped characteristics. The capability can recover if the current density returns from 1.0 A/g to 0.1 A/g. This means that this loss of capacity is reversible, and there is a maximum capability in the tested range of charge/discharge current density at a sulfurization temperature of 300°C.

To further reveal the relationship of the composition of different phases with the electrochemical performance, EIS is applied to specimens in the initial state (Figure 5). The larger the diameter of the semicircle, the more difficult the migration of the lithium ion at the interface. The shallower the slope, the greater the barrier to lithium-ion diffusion inside the electrodes [25]. As shown in Figure 5(a), the diameter increases and the slope for specimens of pure Zn decreases with increased cycling, suggesting that it is more difficult for lithium ions both to enter the electrode and to migrate within.

The equivalent circuit (inset, Figure 4(b)) matches that in an actual battery because the corresponding fitting curves are completely consistent with those measured. This is attributable to the influences of the sulfurization temperature on the composition and phase of the ZnS materials. When vulcanized at 250°C and 300°C, the slope of the linear portion of the sample is greater, which is due to a higher cubic *β*-ZnS content. Compared with the dense hexagonal *α*-ZnS, the lattice gap of *β*-ZnS is greater and the lithium-ion conductivity is better. The semicircle diameter in the high-frequency region increases with increasing vulcanization temperature; the difficulty of lithium-ion migration at the interface increases due to the increase in the amount of hexagonal *α*-ZnS phase with its lower ionic conductivity.

## 4. Conclusions

A zinc precursor was prepared by DC arc plasma method, then sulfurized at different temperatures to obtain Zn/ZnS composite powders. The microstructure and electrochemical properties of the Zn/ZnS materials with varying degrees of vulcanization were investigated. With increasing sulfurization temperature, pure Zn gradually changes into cubic *β*-ZnS and then cubic *β*-ZnS into hexagonal *α*-ZnS. The cycling performance gradually increases to a maximum at 300°C, declining thereafter. The capability of the ZnS vulcanized at 300°C is maintained at 232.1 mAh/g after 300 cycles under conditions involving a 500 mA/g charge/discharge current density. Diffusion migration of lithium ions is easier in the cubic *β*-ZnS, as confirmed by electrochemical impedance spectroscopy. Furthermore, ZnS nanoparticles present good optical properties and have potential applications in biological tagging and cell imaging.

## Figures and Tables

**Figure 1:** (a) SEM image of the ZnS materials at the sulfurization temperature of 350°C and (b) the corresponding EDX spectra.

**Figure 2:** XRD spectra of the ZnS materials at different sulfurization temperatures.

**Figure 3:** (a) FTIR spectra of ZnS and (b) UV spectrum of ZnS at 350°C.

**Figure 4:** (a) Rate capability and (b) the average specific capacity of the ZnS materials vulcanized at various temperatures.

**Figure 5:** (a) EIS of Zn. (b) EIS and the corresponding equivalent analogue circuits of the ZnS materials at different sulfurization temperatures.

**Table 1:** Cycle performance of Zn/ZnS materials prepared at various sulfurization temperatures.

Temperature (°C)	First discharge capacity (mAh/g)	First charge capacity (mAh/g)	Discharge capacity after 300 cycles (mAh/g)	Retention ratio after 300 cycles (%)
25 (pure Zn)	527.8	405.3	<81.3	<15.4
200	627.4	305.1	99.6	16.0
250	894.8	407.6	156.3	17.5
300	998.8	465.2	230.3	23.1
350	1052.0	511.6	96.7	9.2

## Data Availability

Data sharing not applicable to this article as no datasets were generated or analysed during the current study.
